The article "COV-DLS: Prediction of COVID-19 from X-Rays Using Enhanced Deep Transfer Learning Techniques" was published in 2022. Journal: J Healthc Eng.

# COV-DLS: Prediction of COVID-19 from X-Rays Using Enhanced Deep Transfer Learning Techniques

**DOI:** 10.1155/2022/6216273

**Published:** 2022-04-11

**Authors:** Vijay Kumar, Anis Zarrad, Rahul Gupta, Omar Cheikhrouhou

**Affiliations:** ^1^National Institute of Technology, Hamirpur, Himachal Pradesh 177005, India; ^2^University of Birmingham, Dubai, UAE; ^3^CES Lab, National School of Engineers of Sfax, University of Sfax, Sfax 3038, Tunisia; ^4^Higher Institute of Computer Science of Mahdia, University of Monastir, Mahdia 5111, Tunisia

## Abstract

In this paper, modifications in neoteric architectures such as VGG16, VGG19, ResNet50, and InceptionV3 are proposed for the classification of COVID-19 using chest X-rays. The proposed architectures termed “COV-DLS” consist of two phases: heading model construction and classification. The heading model construction phase utilizes four modified deep learning architectures, namely Modified-VGG16, Modified-VGG19, Modified-ResNet50, and Modified-InceptionV3. An attempt is made to modify these neoteric architectures by incorporating the average pooling and dense layers. The dropout layer is also added to prevent the overfitting problem. Two dense layers with different activation functions are also added. Thereafter, the output of these modified models is applied during the classification phase, when COV-DLS are applied on a COVID-19 chest X-ray image data set. Classification accuracy of 98.61% is achieved by Modified-VGG16, 97.22% by Modified-VGG19, 95.13% by Modified-ResNet50, and 99.31% by Modified-InceptionV3. COV-DLS outperforms existing deep learning models in terms of accuracy and F1-score.

## 1. Introduction

The first known case of the novel coronavirus disease 2019 (COVID-19) appeared in the Wuhan province of China in December 2019. Within months, it had spread across the world. The World Health Organization (WHO) declared the COVID-19 outbreak a “Public Health Emergency of International Concern” on January 30, 2020. On March 11, 2020, the situation was declared a pandemic. As of January 13, 2022, the total global number of confirmed cases was 317,700,427, with 5,531,439 deaths [1]. COVID-19 has affected every region of the world, with confirmed cases in North America (75,618,797), Europe (99,973,414), Asia (88,253,001), South America (41,947,867), Africa (10,337,444), and Oceania (1,569,183) [1, 2].

COVID-19 impacts people in many different ways. The most frequent symptoms are fever, dry cough, and fatigue [3]. Less common symptoms include aches, pains, sore throat, diarrhea, conjunctive, headache, loss of taste or smell, a rash on the skin, and a change in the color of fingers or toes. To contain outbreaks of COVID-19, infected persons must be quarantined; if an infected person is not isolated, they may infect other people. Thus, isolation or quarantine is an effective way to prevent the spread of this virus.

The article "COV-DLS: Prediction of COVID-19 from X-Rays Using Enhanced Deep Transfer Learning Techniques" was published in 2022. Journal: J Healthc Eng.

Various tests such as RT-PCR and RAT are used to determine whether a person is infected; however, they are very costly and time-consuming. To overcome these challenges, radiological imaging techniques can be utilized. Well-known imaging techniques include computed tomography (CT) scans and X-rays of the chest. X-ray images are less expensive than CT scans and are more easily available [4]. X-rays can show the affected part of the body, such as the lungs, as well as infection, pneumonia, tumors, and other conditions. With these benefits, X-ray images can also be used to predict cases of COVID-19. When a person is infected, the virus also attacks the lung. Thus, by using a chest X-ray, we can classify a person as either infected or not infected. By using deep transfer learning techniques and a pretrained model, X-ray images can be classified as “COVID-19” or “normal” [5]. In transfer learning, all related information is collected, and this knowledge is “transferred” to solve various other problems [6]. A deep learning (DL) model can be introduced by taking a data set of X-ray images of the human chest.

The above facts motivated us to design a transfer learning technique for the classification of COVID-19 using chest X-ray images. In this paper, novel deep transfer learning techniques termed “COV-DLS” are proposed for discriminating coronavirus infection in chest X-ray images. COV-DLS consists of two phases: heading model construction and classification. The heading model construction phase utilizes four modified deep learning architectures, namely Modified-VGG16, Modified-VGG19, Modified-ResNet50, and Modified-InceptionV3. The output of these modified models is applied during the classification phase. The main contributions of this paper are as follows:

1. Four transfer learning models, namely VGG16, VGG19, ResNet50, and InceptionV3, are modified for COVID-19 classification.
2. The average pooling layer, one dense layer with ReLU, dropout, and one dense layer with softmax are incorporated in the original deep learning architectures for further refinement. The dropout layer is used to prevent the overfitting problem. The average pooling layer is used to smooth the image.
3. Modified deep learning architectures (i.e., Modified-VGG16, Modified-VGG19, Modified-ResNet50, and Modified-InceptionV3) are tested on a chest X-ray data set and achieved better efficiency than their original versions.
4. Modified-InceptionV3 is compared with ten well-known deep learning models and is found to achieve better accuracy and F1-score than the other models.

The article "COV-DLS: Prediction of COVID-19 from X-Rays Using Enhanced Deep Transfer Learning Techniques" was published in 2022. Journal: J Healthc Eng.

The remaining structure of this paper is as follows.  Section 2 presents the related work done in the field of COVID-19. The concepts of convolutional neural networks and transfer learning are discussed in Section 3. The proposed modifications in deep learning architectures are presented in Section 4. Experimental results and discussion are mentioned in Section 5, followed by the conclusion in Section 6.

## 2. Related Work

For many years, DL has been widely used in various spheres of industry, such as natural language processing (NLP), video recognition, medical science, and entertainment. In the field of medical science, it has been very useful in predicting and diagnosing diseases such as tumors, pneumonia, and cancer. This technique is now being used to identify COVID-19 from X-ray images. This is achieved by using convolutional neural networks (CNN) and transfer learning to optimize the pretrained models and enhance their performance in identifying COVID-19 from X-ray images.

Researchers have been working extensively in this field to predict COVID-19 patients by using many DL models. Alshazly et al. [3] modified two DL models, ResNet and DenseNet, to classify COVID-19 and normal patients with 93.87% accuracy for 2-class and 83.89% accuracy for 3-class. Zhang et al. [4] introduced a novel anomaly detection model based on DL for achieving fast and reliable screening. This model consisted of three major components: a backbone network, a classification head, and an anomaly detection head. It was trained by using stochastic gradient descent with several useful parameters. The sensitivity for the proposed model was 96%, and specificity was 70.65%. Makris et al. [5] developed a DL model to identify COVID-19 patients from chest X-rays; convolutional neural networks (CNN) were utilized in this model. Alazab et al. [6] developed an AI-based technique for the prediction and detection of COVID-19 in patients. The prophet algorithm (PA), autoregressive integrated moving average (ARIMA) model, and long short-term memory neural network (LSTM) were incorporated into the proposed model. The accuracy of the prediction results was 94.8% and 88.43% in Australia and Jordan, respectively. The major benefit of AI is that it can be implemented to categorize unseen images.

To diagnose pneumonia-afflicted patients, Narin et al. [7] constructed multiple pretrained CNN models that operate on X-ray images following the ResNet50, ResNet101, ResNet152, InceptionV3, and Inception-ResNetV2 models. Classifications of the processed images were split into four groups—COVID-19, normal, viral pneumonia, and bacterial pneumonia—and further subjected to 5 fivefold cross-validations. The highest accuracy was obtained by ResNet50 at 98%. Using a DL algorithm, Sethy et al. [8] extracted features from chest X-ray images, using them with SVM to determine whether the patient was infected or normal. Thirteen different CNN models were used to achieve 95.38% accuracy by using ResNet50 and SVM. Minaee et al. proposed a model prepared on 5,000 X-ray images (2,000 for training and 3,000 for testing) for the detection of COVID-19. Transfer learning was used to predict COVID-19 patients with the help of ResNet18, ResNet50, SqueezeNet, and DenseNet-121, achieving a sensitivity rate of around 98% and a specificity rate of around 90%. Ozturk et al. [9] proposed a model that can provide accurate diagnostics for binary classification (COVID-19 vs. no-findings) and multiclass classification (COVID-19 vs. no findings vs. pneumonia). This model produced a classification accuracy of 98.08% in the case of binary classes and 87.02% in the case of multiclass cases. The DarkNet model was used for classification in the “you only look once” (YOLO) real-time object detection system but has only a limited number of COVID-19 X-ray images. Apostolopoulos and Mpesiana [10] differentiated between bacterial pneumonia, confirmed COVID-19 disease, and normal results using network architecture transfer learning.

The article "COV-DLS: Prediction of COVID-19 from X-Rays Using Enhanced Deep Transfer Learning Techniques" was published in 2022. Journal: J Healthc Eng.

With transfer learning, different abnormalities can be easily recognized in small data sets of medical images. Singh et al. [11] used chest CTs to differentiate an infected person from a non-COVID-19-infected person by using multiobjective differential evolution (MODE) based on CNN. Adhikari [12] presented a network called “automatic diagnosis medical analysis for the COVID-19 detection system” (ADMCDS). This network identifies the most infected part of the lungs by taking the input of both types of images (i.e., X-rays and CT scan images). Singh et al. [13] used the deep forest model to identify the early detection of COVID-19. The ensemble learning was utilized in the proposed model. Their model attained greater accuracy than the existing models.

Khan et al. [14] proposed a model named CoroNet, based on Xception architecture, to differentiate COVID-19 chest X-rays from bacterial pneumonia, viral pneumonia, and normal chest X-rays with an accuracy of 98%. Ghoshal and Tucker [15] utilized the drop-weights-based Bayesian CNN model for the detection of COVID-19 from X-ray images and achieved an accuracy of 89.60%. Elbishlawi et al. [16] developed a Corona-Net model to recognize COVID-19 from X-ray images, which utilized the concepts of both encoder and decoder networks. The accuracy obtained from Corona-Net is 95%. Uçar and Korkmaz [17] used the SqueezeNet model with Bayesian optimization to predict COVID-19 from X-ray images. Asif et al. [18] proposed a model using deep CNN to identify coronavirus pneumonia-infected patients by using chest X-ray images and attained an accuracy of more than 98%. Sahinbas and Catak [19] applied CNN models, namely VGG16, VGG19, ResNet, DenseNet, and InceptionV3, to detect COVID-19 in X-ray images. The highest accuracy was 80%, achieved by VGG16.

The article "COV-DLS: Prediction of COVID-19 from X-Rays Using Enhanced Deep Transfer Learning Techniques" was published in 2022. Journal: J Healthc Eng.

Wang et al. [20] developed a COVID-19 detection technique based on the concept of discrimination- and localization-based deep learning techniques; the former was used to extract the lung features from the chest X-ray images, after which the latter was trained on the extracted lung features and localized the region of interest in the lungs. This method attained better accuracy than the other techniques. Chen et al. [21] designed a coronavirus detection algorithm using ResNet18 to extract the features from chest X-ray images. A metaheuristic algorithm was then used to optimize the extracted features, which were then applied on a support vector machine for COVID-19 classification. This approach was able to differentiate the presence or absence of COVID-19 from chest X-ray images.

Oulefki et al. [22] proposed an automatic coronavirus detection technique using chest CT images. They modified the local contrast enhancement technique for detecting the detailed CT scan image. Next, the lung image region was segmented into small subregions. Their proposed technique achieved better results than the existing classical and deep learning techniques, and it can be further enhanced by using the segment of ground-glass opacity. Liu et al. [23] developed a weekly supervised technique for COVID-19 classification. An uncertainty-based teacher framework was utilized for model training. The developed technique was tested on three different data sets and achieved better performance measures than the existing deep learning architectures. The performance of this method can be further enhanced through the concept of noise annotations. He et al. [24] presented an adversarial framework for discriminating COVID-19-infected patients using chest CT images. Three mutation operators were used to modify the generator for segmentation, and a gradient penalty was used to eliminate gradient vanishing. The proposed method was tested on four different data sets and attained 0.42% and 0.48% improvements in dice similarity coefficient and structure measure, respectively.

It is observed in the extant literature that the existing models are able to identify COVID-19 from chest X-ray images. However, these models' performance is still far from optimal.

The article "COV-DLS: Prediction of COVID-19 from X-Rays Using Enhanced Deep Transfer Learning Techniques" was published in 2022. Journal: J Healthc Eng.

## 3. Background

In this section, the preliminary concepts of deep transfer learning architectures are discussed.

### 3.1. Convolutional Neural Network (CNN)

CNN can be used to detect objects and faces, as well as in video recognition. The architecture of CNN was an inventiveness of the visual cortex [25, 26]. There are three layers in CNN architecture: the convolution layer, the pooling layer, and the fully connected layer. The model proposed in this study can learn through the convolutional and pooling layers. Classification can be done with the help of a fully connected layer [26].

To train and test CNN models, every input image passes through the convolutional, pooling, and fully connected layers. Next, a softmax activation function was used to categorize the images with probabilistic values between 0 and 1 [27].  Figure 1 describes the architecture of CNN.

The function of the convolution layer is to extract the attributes from the input image. The convolution operation is a type of mathematical operation performed on an input image and filter or kernel matrix to obtain the feature map [28].

Let us assume that the image has the size of (*h*1 × *w*1 × *d*1), where *h*1 represents height, *w*1 represents width, and *d*1 represents depth. A kernel (filter) of the dimension is (*h*2 × *w*2 × *d*2). After performing the convolution operation between them, the dimensional output is (*h*3 × *w*3 × *d*2).  Figure 2 shows the multiplication operation between the image and kernel matrix.

The pooling layer plays a vital role by reducing the total number of dimensions (or parameters) and maintaining the main features. The different categories of pooling are max pooling, min pooling, and mean pooling. In max pooling, the max pixel is selected from an image based on pool size. The fully connected layers are present at the edge of the neural network to classify the images with the help of the sigmoid activation function [28]. This layer is also known as a “feed-forward neural network” [29]. A fully connected layer takes input from the output of the final pooling after flattening. A fully connected network is depicted in Figure 3.

### 3.2. Transfer Learning

Transfer learning collects the knowledge gained during learning and applies it to another problem by transferring that knowledge. In deep learning, various pretrained models are trained on well-defined various data sets; thus, by using these models, better accuracy can be achieved even if the data set is small. This is the researchers' preferred approach [30].

Pan and Yang conducted an extensive survey on transfer learning [31]. They found that in the transfer learning process, the learning procedure did not start at the beginning; rather, it began with the knowledge collected to solve another task. As a result, we can see that transfer learning involves two things: using the previously accumulated knowledge and ignoring the imperative to start the learning process from scratch. By doing these two things, the process was observed to be both quicker and more accurate [32].

The article "COV-DLS: Prediction of COVID-19 from X-Rays Using Enhanced Deep Transfer Learning Techniques" was published in 2022. Journal: J Healthc Eng.

In deep learning, transfer learning allows the preliminary preparation of the CNN to be done on large-scale training data sets. Through such training, the CNN model learns all the necessary features of the image data. This availability of data is the initial component required to train the model well. Finally, this model is tested to recognize and categorize various images; the results of this testing are used to determine whether the model is suitable for transfer learning.

#### 3.2.1. VGG Architecture

VGGNet architecture was designed and developed by Simonyan and Zisserman in 2014 [33]. VGG stands for Visual Geometric Group, and it is a CNN architecture. This is a simple model, so the basic difference between this VGG and previous models lies in its in-depth structure and in having the end layers associated with two or three convolution layers. As a result, this VGG model is widely used in CNN [33]. VGG network architecture is very large, with nearly 138 million parameters [34]. This model is trained using millions of images and collects the important features and information of 1,000 different categories from the ImageNet data set (see Figure 4).

In VGG-16 architecture, “16” represents several layers that have weights, of which 13 are convolution layers and 3 are convolution filters. Every convolution layer comprises a ReLU activation function and max pooling layers for sampling. Ultimately, this architecture consists of three fully connected layers that are used for categorization. Of the three, two work as hidden layers, and the last is used for the classification of 1,000 image categories in the ImageNet Database [33]. VGG-16 always uses filters of 3 ∗ 3 with a stride of 1 in the convolution layer and uses a SAME padding layer 2 ∗ 2 with a stride of 2. It works well for both object classification and edge detection problems [34].

VGG-19 architecture is the same as VGG-16 architecture; it differs only by having 19 layers with trainable weights, among which there are 16 CNN layers and 3 fully connected layers.

#### 3.2.2. ResNet Architecture

ResNet stands for “residual network.” This architecture is designed to be much more comprehensive and deeper than earlier similar architectures. This network was proposed in 2015 by He et al. [35]. It achieved first place in an ImageNet contest held in 2015, with a very low rate of error at 3.6% [35].

The article "COV-DLS: Prediction of COVID-19 from X-Rays Using Enhanced Deep Transfer Learning Techniques" was published in 2022. Journal: J Healthc Eng.

To solve a complex problem, some architectural layers can be appended to increase performance and accuracy. In general, the number of layers is increased to reduce the error rate, but at a certain point, a common problem, known as the “vanishing/exploding gradient,” occurs. ResNet architecture overcomes this problem by introducing skip connections or identity shortcut connection techniques. This configuration essentially bypasses the training for some layers and is therefore directly connected to the output [33]. The residual block is depicted in Figure 5.

This network employs layer mapping instead of layers; such mapping is called “residual mapping.” As we can see, residual mapping, *H*(*x*) = *F*(*x*) + *x*, comes from initial mapping, *H*(*x*) = *F*(*x*). The benefit of this configuration is that if a given layer downgrades the performance of the architecture, then that layer is automatically bypassed by regularization, thereby resolving the vanishing/exploding gradient problem.

ResNet50 is a variation of the ResNet model consisting of 50 layers (48 convolution layers, 1 maxpooling, and 1 average pooling layer). The ResNet50 model performs simple training and has many advantages due to its capacity for residual learning directly from images rather than image features [35]. Thus, it is not necessary to first extract the features before training the model.

#### 3.2.3. InceptionV3 Architecture

The InceptionV3 model is used to identify images and recognize objects. It has an accuracy of about 78.1%, and its low error rate on the ImageNet data set in 2015 secured second place for image categorization in ILSVRC. Szegedy et al. [36] describe four versions of inception in its architecture. It has 42 layers, rendering it superior to VGGNet [37] while costing 2.5 times more than GoogleNet [38].

## 4. Proposed Technique

In this study, we used the publicly available data set of COVID-19 X-ray images [39, 40]. Because these X-ray images were available in different sizes and resolutions, we uniformly resized them to 224 × 224. Because the amount of data is reduced at this size, we applied image augmentation. For this paper, we prepared a head model and added the pretransfer learning models such as VGG16, VGG19, ResNet50, and InceptionV3 to achieve results on the accuracy, precision, recall, and the loss and accuracy graph. The proposed model is inspired by the work done by Sahinbas and Catak [19].  Figure 6 shows the architecture of the proposed model, and its steps are described below:

Step 1: Image acquisition
Initially, X-ray images of COVID-19 and non-COVID-19 patients were collected from publicly accessible sites such as GitHub [39] and Kaggle [40].
Step 2: Update data
After loading the data set, we extracted the labels and collected them. All the images were converted from BGR to RGB channels and then resized to 224 × 224.
Step 3: Perform one-hot encoding
One-hot encoding was performed on the labels using LabelBinarizer, which is a class of Scikit-Learn that takes input as categorical data and returns a NumPy array [41].
Step 4: Data set splitting and augmentation
In this step, the data set was split into “train” and “test” parts of 80% and 20%, respectively, and we initialized the data augmentation object with parameters such as rotation range at 15 and fill mode initialized as “nearest.” There are various types of fill modes, such as “constant,” “nearest,” “reflect,” and “wrap.”
Step 5: Initialize the base model
Next, we initialized the base model with various pretrained models such as VGG16, VGG19, ResNet50, and InceptionV3. However, neither the top nor the head of the model was loaded.
Step 6: Construct the model head
In this step, we built the head of the base model and appended it to the top of the model.
  - The head model begins with the output of the root/base model
  - Average pooling of size 4 × 4 is applied
  - Next, the head model is flattened
  - The dense layer of 64 is applied on the head model with the activation function “ReLU”
  - Dropout layer with a rate of 0.5 is applied on the head model to prevent overfitting
  - Finally, a dense layer of size 2 is applied because of binary classification with a softmax activation function
As the head model was prepared, the base model was placed at the bottom with the head model on top of it. The complete model was then ready to train.
Step 7: Compile the model
Next, the model was compiled with the Adam optimizer, which is a combination of AdaGrad and RMSProp algorithms that provides better optimization of noisy data [15]. The initial learning rate chosen was 0.001.
Step 8: Train the model
The model was trained with 25 epochs and 32 batch sizes on 80% of the data.
Step 9: Test the model
Next, the model was tested on the remaining 20% of the data set and achieved the required results for accuracy, recall, F1-score, specificity, sensitivity, and so on. With the help of these results, we plotted the loss and accuracy graph.

The article "COV-DLS: Prediction of COVID-19 from X-Rays Using Enhanced Deep Transfer Learning Techniques" was published in 2022. Journal: J Healthc Eng.

## 5. Materials and Method

### 5.1. Data Set

For this investigation, the chest X-ray images of COVID-19 patients and normal patients were used. The data sets for COVID-19 and normal patients are publicly available on the GitHub repository [39] and on Kaggle [40], respectively. In this model, chest X-ray images were used to classify the images as “COVID-19” or “normal.” A total of 720 chest X-ray images were used, of which 540 were of normal lungs and 180 were of lungs affected by COVID-19. The data set was divided into 80% for training and 20% for testing. All the X-ray images were different in shape and size. All the images were resized to 224 × 224.

Image augmentation was used to increase the sample numbers to improve the model's performance in classifying the images. Our image augmentation parameters had the rotation range set to 15 and the fill mode kept as “nearest.” Figure 7 illustrates sample chest X-ray images.

### 5.2. Experimental Setup

For this work, an experiment has been performed with the help of Google Colab, which is an open-source IDE for Python code. The advantage of using Google Colab's predefined libraries (such as NumPy, Pandas, Matplotlib, Seaborn, Tensorflow, and Keras) is that they are easy to use and their methods, and functions can be used to solve complex problems relatively straightforwardly.

Table 1 contains all of the parameters and information used to prepare the model and provide the experimental results:

### 5.3. Performance Metrics

Because we know that this data set is balanced except for the optimal classifier, having only one result to determine accuracy is not enough. We therefore used other metrics such as precision, recall, and F1-score. These four metrics are ordinary measurements used in machine learning for the analysis of classification [42–44].

The above-mentioned metrics are evaluated with the help of a confusion matrix using four terminologies: true positive (TP), false positive (FP), true negative (TN), and false negative (FN). All the metrics are defined below:

(1) $$\begin{array}{c} \text{precision}=\frac{\text{TP}}{\text{TP}+\text{FP}}, \end{array}$$

(2) $$\begin{array}{c} \text{recall}=\;\frac{\text{TP}}{\text{TP}+\text{FN}}, \end{array}$$

(3) $$\begin{array}{c} F1-\text{score}=\frac{2\times \text{precision}\times \text{recall}}{\text{precision}+\text{recall}}, \end{array}$$

(4) $$\begin{array}{c} \text{accuracy}=\frac{\text{TP}+\text{TN}}{\text{TP}+\text{TN}+\text{FP}+\text{FN}}. \end{array}$$

### 5.4. Results and Discussion

Table 2 shows the performance results for each transfer model in identifying COVID-19. Various models have yielded different results, and maximum accuracy was achieved by the Modified-VGG16 and Modified-InceptionV3 models. With the help of a confusion matrix, we achieved the other metrics of precision, recall, F1-score, sensitivity, and specificity.

“Precision” describes the percentage of actual positive results out of the total positive (TP + FP) predicted by the model. “Recall” is defined as the total number of true positives out of the total positive value. Equations (1) and (2) represent precision and recall, respectively. F1-score is calculated as a harmonic mean between precision and recall, as defined in equation (3). “Accuracy” can be determined by assessing the extent of correct prediction among all values, and it is represented in equation (4). “Sensitivity” (also known as “true positive rate”) is an effective way to determine true positives from all available classes. Similarly, “specificity” is an effective way to determine true negatives from all available classes.

The article "COV-DLS: Prediction of COVID-19 from X-Rays Using Enhanced Deep Transfer Learning Techniques" was published in 2022. Journal: J Healthc Eng.

The figure below exhibits the confusion matrix of each transfer learning model where 0 indicates COVID-19 and 1 denotes normal.

Figure 8 shows the confusion matrix of different models used to predict the above performance metrics. With the help of a confusion matrix, we can predict the values of TP, TN, FP, and FN. True/false represents actual values whereas positive/negative represents the predicted values.

In the above confusion matrices, 1 represents COVID-19 X-rays, and 0 represents normal X-rays. These matrices were computed based on our 20% data set, and by using its values, all other metrics (such as precision, recall, F1-score, sensitivity, and specificity) were computed.

#### 5.4.1. Accuracy and Loss

Accuracy and loss graphs are also plotted for all four models: Modified-VGG16, Modified-VGG19, Modified-ResNet50, and Modified-InceptionV3. Figures 9 and 10 show the accuracy and loss curves obtained from the proposed Modified-VGG16, Modified-VGG19, Modified-ResNet50, and Modified-InceptionV3 models, respectively.

Figures 9 and 10 show the accuracy versus loss graphs for each modified model. Here, the *x*-axes show the number of epochs, and the *y*-axes show accuracy/loss. In the above graphs, the training as well as the validation of the models are plotted. The best results are achieved by Modified-InceptionV3.

#### 5.4.2. Comparative Analysis

The performance of four modified deep learning architectures (i.e., VGG16, VGG19, ResNet50, and InceptionV3) is compared with that of their existing, unmodified models.  Figure 11 depicts the comparative analysis of modified deep learning architectures and original deep learning architectures in terms of accuracy, precision, recall, and F1-score. It can be seen in the figures below that the modified proposed architectures performed better than the original architectures. Furthermore, it can be seen from Figure 11 that among the modified architectures, Modified-InceptionV3 performed best.

The performance of Modified-InceptionV3 is compared with 10 well-known deep learning-based COVID-19 detection models, namely: COVID-Xpert [45], COVID-Net [46], COVID-Caps [47], COVID-ResNet [48], Corona-Net [16], DarkNet [9], ShuffleNet [8], GoogleNet [8], DenseNet201 [8], and MobileNetV2 [8].  Figure 12 shows the comparative analysis of these models in terms of accuracy. Modified-InceptionV3 achieves an accuracy measure of 0.9931, thus outperforming the existing deep learning models. DarkNet is the second-best model, followed by Corona-Net in third place.

The article "COV-DLS: Prediction of COVID-19 from X-Rays Using Enhanced Deep Transfer Learning Techniques" was published in 2022. Journal: J Healthc Eng.

Figure 13 illustrates the performance comparison between Modified-InceptionV3 and the existing deep learning models in terms of F1-score. It is observed from the figure that the F1-score obtained from Modified-InceptionV3 is better than that of the other models. The F1-score values obtained from Modified-InceptionV3 and DarkNet are 0.99 and 0.96, respectively. F1-scores obtained from Corona-Net and COVID-ResNet are 0.94 and 0.93, respectively.

## 6. Conclusion and Future Work

This study analyzes the classification of COVID-19 positive and normal patients through the analysis of X-ray images. In this paper, four pretrained models (i.e., VGG16, VGG19, ResNet50, and InceptionV3) have been modified. Dense and average pooling layers have been incorporated in the original architectures for further refinement, and the modified architectures have been tested on a chest X-ray data set. Data augmentation has been performed to increase the data set's size. Modified-InceptionV3 yielded the greatest accuracy at 99.31%. Modified-VGG16, Modified-VGG19, and Modified-ResNet50 yielded accuracy measures of 98.61%, 97.22%, and 95.13%, respectively. The modified pretrained models achieved better results than their original models. Modified-InceptionV3 has also been compared with 10 well-known deep learning models, all of which it outperforms in terms of accuracy and F1-score.

This data set consisted of a limited number of images; it follows that greater accuracy can be achieved by increasing the number of X-ray images. Alternatively, to achieve greater accuracy, pretrained models can be assembled. Through such assembly and by increasing the data set, not only accuracy—but also other results such as precision, recall, F1-score, sensitivity, and specificity—can be increased. In future research, new techniques or models can be used to further enhance performance.

## Figures and Tables

**Figure 1:** CNN architecture.

**Figure 2:** Multiplication between image matrix and kernel.

**Figure 3:** Fully connected network.

**Figure 4:** VGG-16 architecture.

**Figure 5:** Residual block.

**Figure 6:** Proposed deep learning architecture.

**Figure 7:** X-ray sample images: (a) COVID-19 X-ray and (b) normal X-ray.

The article "COV-DLS: Prediction of COVID-19 from X-Rays Using Enhanced Deep Transfer Learning Techniques" was published in 2022. Journal: J Healthc Eng.

**Figure 8:** Confusion matrix of different transfer models: (a) Modified-VGG16, (b) Modified-VGG19, (c) Modified-ResNet50, and (d) Modified InceptionV3.

**Figure 9:** Accuracy graphs of different models: (a) Modified-VGG16, (b) Modified-VGG19, (c) Modified-ResNet50, and (d) Modified-InceptionV3.

**Figure 10:** Loss graphs of different models: (a) Modified-VGG16, (b) Modified-VGG19, (c) Modified-ResNet50, and (d) Modified-InceptionV3.

**Figure 11:** Performance comparison between the existing and modified deep learning architecture: (a) VGG16 versus Modified-VGG16, (b) VGG19 versus Modified-VGG19, (c) ResNet50 versus Modified-ResNet50, and (d) InceptionV3 versus Modified-InceptionV3.

**Figure 12:** Accuracy comparison of Modified-InceptionV3 versus existing deep learning models.

**Figure 13:** F-1 score comparison of Modified-InceptionV3 versus existing deep learning models.

**Table 1:** Parameters and information required for the experiment.

Information	Value
Type of data set	X-ray images
Size of data set	720 (normal: 180; COVID-19: 540)
Size of training and testing data	Train: 80%; test: 20%
Models	VGG16, VGG19, ResNet50, InceptionV3
Learning rate	0.001
Optimizer	Adam
Activation functions	ReLU and softmax
Dropout	0.5
Metrics	Accuracy, precision, recall, sensitivity, specificity, F1-score
Graph	Loss and accuracy graph

**Table 2:** Performance results of each transfer model for COVID-19 identification by the proposed model.

Model	Accuracy	Precision	Recall	F1-score	Sensitivity	Specificity
Modified-VGG16	0.9861	0.97	0.97	0.97	0.97	0.99
Modified-VGG19	0.9722	0.97	0.92	0.94	0.92	0.99
Modified-ResNet50	0.9513	0.94	0.86	0.89	0.86	0.98
Modified-InceptionV3	0.9931	1.00	0.97	0.99	0.97	1.00

## Data Availability

No data were used to support this study
